The article "Bioinformatics Methods Reveal the Biomarkers and the miRNA-mRNA Network in Hepatocellular Carcinoma" was published in 2022. Journal: J Healthc Eng.

# Bioinformatics Methods Reveal the Biomarkers and the miRNA-mRNA Network in Hepatocellular Carcinoma

**DOI:** 10.1155/2022/9963096

**Published:** 2022-03-16

**Authors:** Yang Liu, Haoliang Zhang, Xue Han, Xiaowei Xing

**Affiliations:** ^1^Department of Oncology, Tangshan Workers' Hospital, Tangshan City 063000, Hebei Province, China; ^2^Department of Cardiovascular Internal Medicine, Tangshan Workers' Hospital, Tangshan City 063000, Hebei Province, China

## Abstract

Hepatocellular carcinoma (HCC) has threatened the health of humans, and few therapeutic strategies can completely uproot this illness. Bioinformatics methods have been widely used for investigating the pathological mechanisms of disease. In this study, datasets including GSE20077 and GSE108724, obtained from the Gene Expression Omnibus (GEO) database, were used for investigating the biomarker and molecular mechanism of HCC. The differentially expressed genes (DEGs) in the datasets were identified, and the targets of the miRNAs were searched in the miRDIP and miRNET databases. Enrichment analysis was performed for delving the molecular mechanism of DEGs, and protein-protein interaction (PPI) networks and miRNA-mRNA networks were used to reveal the hub nodes and the related interaction relationships. Moreover, the expression and diagnostic values of hub nodes were analyzed with the GEPIA2 database. The results showed that 53 upregulated miRNAs and 48 downregulated miRNAs were found in GSE20077, and 55 upregulated miRNAs and 69 downregulated miRNAs were found in GSE108724. Moreover, seven common miRNAs including miR-146b-5p, miR-338-3p, miR-375, miR-502-3p, miR-532-3p, miR-532-5p, and miR-557 were found in the datasets. The targets of the common miRNAs were related with the P53, HIF1, Wnt, and NF-*κ*B pathways. Besides, YWHAZ and CDC42 were identified as the hub nodes and served as the downstream targets of miR-375-3p. The GEPIA2 database showed that YWHAZ and CDC42 were related with the survival rate of the patients. In conclusion, this study suggests that miR-375-3p functions as a tumor suppressor which could inhibit the progression of HCC via targeting YWHAZ and CDC42.

## 1. Introduction

Hepatocellular carcinoma (HCC) is a malignant cancer with a high incidence and mortality [1]. Statistically, more than 800000 people have been diagnosed with HCC in the world in 2018 [2]. HCC is characterized by poor prognosis and low survival rates. At present, surgery, radiotherapy, and chemotherapy are still major strategies for HCC treatment in early stages [3, 4]. However, considerable patients are in the advanced stage when they first accept the diagnosis. The current therapeutic techniques can partly improve the symptoms of HCC, while the prognosis and long-term survival rates of the patients remain unsatisfactory [5, 6]. Although many researchers have focused on the pathological mechanism of HCC and increasing biomarkers have been excavated for clinical use, the molecular mechanism of this disease has not been illustrated thoroughly [7, 8]. Therefore, more research studies are still necessary for illustrating the pathological mechanism of this disease.

MicroRNAs (miRNAs), an endogenous noncoding RNA with a single-strand, play great roles in cellular metabolism including the cell cycle, differentiation, and so on [9]. In recent decade, increasing numbers of reporters have indicated that miRNA dysfunction is involved in the development of various diseases, and some miRNAs have been identified as biomarkers which have been applied in clinical diagnosis and treatment [10, 11]. For HCC, miRNA dysfunction also serves as a critical role which can induce the malignant behaviors of the tumor cells [12]. Although considerable research studies have revealed the roles and molecular functions of some miRNAs in the progression of HCC, the global regulation network of miRNAs in HCC remains unclear. Microarray has been widely used to identify disease-related factors and reveal the related pathological mechanism, which could supply valuable references for clinical treatment [13].

In this study, the datasets in the GEO database were used to screen the key factors of HCC, and the related molecular mechanisms of those genes were investigated with bioinformatics methods, providing some references for HCC treatment.

## 2. Materials and Methods

### 2.1. Data Source

The datasets including GSE20077 and GSE108724 were obtained from the Gene Expression Omnibus (GEO) database (https://www.ncbi.nlm.nih.gov). The matrix files of GSE20077 and GSE108724 were obtained by GEO2R, and the raw data of the datasets were downloaded by the GEOquery package of the R language.

### 2.2. Identification of Differentially Expressed Genes

The differentially expressed genes (DEGs) in GSE20077 and GSE108724 were obtained with GEO2R analysis of the GEO database. In brief, the matrix files of GSE20077 and GSE108724 were obtained by the GEO2R tool of the GEO database. For GSE20077, 3 normal primary human liver cell lines and 7 human HCC cell lines were selected for GEO2R analysis. For GSE108724, 7 tumor tissues and 7 normal liver tissues were selected for GEO2R analysis. Moreover, the miRNAs with |logFC| > 1.5 were selected as the DEGs. Moreover, the common genes in GSE20077 and GSE108724 were screened and visualized with the VENNY online tool (https://bioinfogp.cnb.csic.es/tools/venny/index.html).

### 2.3. Enrichment Analysis

The regulation mechanisms of the DEGs in HCC were enriched with the Kyoto Encyclopedia of Genes and Genomes (KEGG) and Gene Ontology (GO) enrichment analysis. In brief, the potential targets of the miRNAs were predicted by the miRDIP (https://ophid.utoronto.ca/mirDIP/index.jsp) and miRNET (https://www.mirnet.ca/) databases, and the common genes were selected as the targets of the miRNAs. The targets were upregulated in the DAVID database, and the KEGG enrichment was performed by the online tools. The pathways with *P* < 0.05 were visualized with ggplot2 of R language. For the differentially expressed miRNAs in HCC, the targets were predicted with the miRDIP database and then used for KEGG enrichment.

### 2.4. GO Enrichment Analysis

The molecular functions of the DEGs were analyzed with GO enrichment analysis. In short, the targets of the miRNAs were uploaded to the DAVID database to obtain the related ENTREZIDs. Moreover, the ENTREZIDs were enriched with the R language. For differentially expressed miRNAs, the targets of the miRNAs were used for GO enrichment analysis.

### 2.5. Network Analysis

The protein-protein interaction (PPI) network and miRNA-mRNA network were used to investigate the regulation mechanism of the DEGs in GSE20077 and GSE108724. In brief, the targets of DEGs were analyzed with the STRING database (https://cn.string-db.org/), and then visualized with Cytoscape. The targets with the highest combined scores were selected as the hub nodes. Moreover, the miRNA-mRNA network was used to exhibit the interaction relationship.

### 2.6. Diagnostic Values Identification

The targets of the miRNAs were analyzed and visualized with the GEPIA2 database (https://gepia2.cancer-pku.cn/#index). In brief, the targets of miRNAs were uploaded to the GEPIA2 database, and the expression and related survival curve of the targets in the clinical samples were analyzed by GEPIA2.

## 3. Results

### 3.1. DEGs Identification

To observe the difference of HCC cells and normal liver cells, the DEGs in GSE20077 and GSE108724 were screened. For GSE20077, 3 normal primary human liver cell lines and 7 human HCC cell lines were selected for GEO2R analysis. For GSE108724, 7 tumor tissues and 7 normal liver tissues were selected for GEO2R analysis. The results showed that 53 upregulated miRNAs and 48 downregulated miRNAs were found in GSE20077, and 55 upregulated miRNAs and 69 downregulated miRNAs were found in GSE108724 (Figure 1 and 2). Moreover, 7 common miRNAs including miR-146b-5p, miR-338-3p, miR-375, miR-502-3p, miR-532-3p, miR-532-5p, and miR-557 were found in GSE20077 and GSE108724.

### 3.2. Functions and Pathways Enrichment Analysis

To investigate the functional modules in the progression of HCC, the targets of the DEGs in GSE20077 and GSE108724 were screened by the miRDIP and miRNet databases and analyzed with GO and KEGG enrichment. The results showed that 924 genes and 1047 genes were screened from miRDIP and miRNet, respectively. Moreover, 185 common targets were selected for GO and KEGG enrichment analysis (Figure 2(a)). The results of GO enrichment showed that the targets of the miRNAs were involved in the process of the transcription (Figure 2(b)). The KEGG enrichment showed that the targets of the miRNAs were related with the P53, HIF1, Wnt, and NF-*κ*B pathways (Figure 2(c)).

### 3.3. Network Analysis

To reveal the molecular mechanism of HCC, the DEGs in GSE20077 and GSE108724 were analyzed with the PPI network and miRNA-mRNA network. The PPI network showed that three clusters were found in the common targets, including cluster 1 with 9 nodes and 34 edges, cluster 2 with 4 nodes and 10 edges, and cluster 3 with 11 nodes and 32 edges. In addition, ERBB2, YAP1, CDH2, and JAG1 were identified as the hub nodes in cluster 1; HIF1A, CDC42, and JAK2 were identified as the hub nodes in cluster 2; and YWHAZ, CRK, and ERBB4 were identified as the hub nodes in cluster 3 (Figure 3(a)–3(c)). Moreover, the miRNA-mRNA network is shown in Figure 3(d). CDC42, JAK2, YAP1, and YWHZ were the targets of miR-375-3p.

### 3.4. The Expression of the Hubs Nodes in HCC

To investigate the diagnostic values of the hub nodes, the expression and survival curves of the hub nodes were analyzed with the GEPIA database. The results showed that increased CDC42, CDH2, ERBB2, JAG1, YAP1, and YWHAZ were found in the tumor tissues (Figure 4). Moreover, it was also found that the abundances of CDC42 and YWHAZ were related with the survival rates of the patients. Those observations suggested that CDC42 and YWHAZ served as the biomarkers in HCC (Figure 5).

## 4. Discussion

HCC is still one of the most dangerous diseases in the world. Even with modern therapeutic techniques, the prognosis of patients with HCC still lacks significant improvement, which is an intractable question for the current medical system [14]. Hence, the treatment for HCC has received continuous attention. In this study, bioinformatics methods were used to reveal the biomarkers and delve into the pathological mechanism of HCC. During this process, the DEGs of the pathological samples and normal samples were identified with the datasets including GSE20077 and GSE108724. The biomarker genes were identified and the molecular interactions of the DEGs were also investigated by PPI and miRNA-mRNA network analysis.

Microarray analysis has been widely used for observing the change of gene expression in cells or tissues, which could directly reflect the mechanism of cellular metabolism [15]. In this study, GSE20077 and GSE108724 were obtained and used for observing the difference of miRNAs profiles in normal and tumor tissues. miRNAs are involved in multiple processes of cellular behaviors ranging from proliferation to apoptosis, which play important roles in cellular activities. In GSE20077 and GSE108724, the miRNA profiling in tumor tissues exhibited significant differences from the normal tissues and seven critical miRNAs including miR-146b-5p, miR-338-3p, miR-375, miR-502-3p, miR-532-3p, miR-532-5p, and miR-557 which may have potential association with the progression of live cancer. miR-146b-5p may serve as an inhibitor role to suppress the aberrant proliferation and invasion of renal cancer cells via blocking the expression of MMP16, while few studies have revealed its role and functions in HCC [16]. In GSE20077 and GSE108724, decreased miR-146b-5p was also found in the tumor tissues, which suggests that miR-146b-5p may function as a tumor suppressor in HCC. Moreover, it was found that miR-338-3p, miR-375, and miR-557 were also remarkably downregulated in the tumor tissues. The research studies have reported that miR-375 can repress the stemness of breast cancer and gastric cancer cells [17, 18]. Wang et al. have indicated that miR-557 upregulation could effectively impede the epithelial-mesenchymal transition and then inhibit the metastasis of osteosarcoma cells [19]. For miR-338-3p, few studies have revealed its role in cancer development; thus, selecting miR-338-3p as a diagnostic biomarker in HCC has to be confirmed by more direct proofs.

Binding mRNAs to restrain the expression of the proteins is one of the critical functions of miRNAs in regulating multiple behaviors of cells [20]. This study also invested the functions of the miRNAs via analyzing their downstream targets. Disorder activation or inactivation of the pathways is a biomarker event in progression. For HCC, considerable studies have confirmed that the malignant progression of the tumor cells is related with dysfunctions of several signaling pathways, such as PI3K/AKT, Wnt/*β*-catenin, and P53 pathways [20–22]. In this study, it was found that the targets of the miRNAs were related with multiple pathways including NF-KB, P53, Wnt, and HIF-1 pathway, and HIF1A, CDC42, and ERBB2 were associated with cancer-related pathways.

In this study, 9 genes including ERBB2, YAP1, CDH2, JAG1, HIF1A, CDC42, JAK2, YWHAZ, and CRK were identified as the hub nodes in the targets of the miRNAs, and CDC42 and YWHAZ were identified to be related with the survival rates of the patients. The study has indicated that CDC42 serves as an oncogene to involve the malignant progression of some tumors [23]. In HCC, upregulated CDC42 has been also found in the tumor cell lines, and CDC42 can also promote the expression of PAK1 to advance the malignant behaviors of the tumor cells [24]. YWHAZ belongs to the 14-3-3 protein family and involves many signal pathways [25]. Aberrant expression of YWHAZ has been observed in various tumors, and it is also associated with the clinical stages of bladder cancer [26]. In HCC, YWHAZ downregulation could also impede the progression of the proliferation and migration of tumor cells [27]. In this study, YWHAZ and CDC42 were found as the downstream targets of miR-375-3p. Moreover, increased ERBB2 and YAP1 were also found in the clinical data of GEPIA2, and they were also identified as the downstream targets of miR-375-3p. Therefore, this study suggests that miR-375-3p plays an inhibitor role in HCC.

## 5. Conclusion

This study suggests that miR-375-3p plays an inhibitory role in HCC progression via targeting the YWHAZ and CDC42.

## Figures and Tables

**Figure 1:** The differentially expressed genes (DEGs) in GSE20077 and GSE108724. (a) Volcano plots of the DEGs in GSE20077. (b) Volcano plots of the DEGs in GSE108724. (c) The common miRNAs in GSE20077 and GSE108724.

**Figure 2:** The molecular functions and the related pathways of the DEGs in GSE20077 and GSE108724. (a) The common targets of the miRNAs in the miRDIP and miRNET database. (b) The GO enrichment analysis of the targets of the miRNAs (MF: molecular function, BP: biological process, and CC: cellular component). (c) The KEGG enrichment analysis of the targets of the miRNAs.

**Figure 3:** Interaction network analysis of the common miRNAs in GSE20077 and GSE108724. ((a–c)) The PPI network analysis for the targets of the miRNAs. (d) The miRNA-mRNA network analysis for the miRNAs and the related targets (miRNA: green and target: orange).

**Figure 4:** The expressions of the targets in tumor tissues originated from the GEPIA2 database. ((a–i)) The expression of CDC24, CDH2, CRK, ERBB2, HIFA, JAG1, JAK2, YAP1, and YWHAZ in the GEPIA2 database.

**Figure 5:** The survival rates of the targets in tumor tissues originated from the GEPIA2 database. ((a–i)) The survival rates of CDC24, CDH2, CRK, ERBB2, HIFA, JAG1, JAK2, YAP1, and YWHAZ in the GEPIA2 database.

## Data Availability

The data to support the findings of this study are available on reasonable request from the corresponding author.
